# Connections between Various Disorders: Combination Pattern Mining Using Apriori Algorithm Based on Diagnosis Information from Electronic Medical Records

**DOI:** 10.1155/2022/2199317

**Published:** 2022-05-13

**Authors:** He Ma, Jingjing Ding, Mei Liu, Ying Liu

**Affiliations:** Department of Medical Records & Statistics, Affiliated Hospital of Xuzhou Medical University, Xuzhou, Jiangsu 221000, China

## Abstract

**Objective:**

Short-term or long-term connections between different diseases have not been fully acknowledged. This study was aimed at exploring the network association pattern between disorders that occurred in the same individual by using the association rule mining technique.

**Methods:**

Raw data were extracted from the large-scale electronic medical record database of the affiliated hospital of Xuzhou Medical University. 1551732 pieces of diagnosis information from 144207 patients were collected from 2015 to 2020. Clinic diagnoses were categorized according to “International Classification of Diseases, 10th revision”. The Apriori algorithm was used to explore the association patterns among those diagnoses.

**Results:**

12889 rules were generated after running the algorithm at first. After threshold filtering and manual examination, 110 disease combinations (support ≥ 0.001, confidence ≥ 60%, lift > 1) with strong association strength were obtained eventually. Association rules about the circulatory system and metabolic diseases accounted for a significant part of the results.

**Conclusion:**

This research elucidated the network associations between disorders from different body systems in the same individual and demonstrated the usefulness of the Apriori algorithm in comorbidity or multimorbidity studies. The mined combinations will be helpful in improving prevention strategies, early identification of high-risk populations, and reducing mortality.

## 1. Introduction

Everyone suffers from multiple kinds of diseases in their whole lives. It is believed that some illnesses can cooccur within a certain period. That is, these disorders may have some sort of connection with each other in the same individual. These connections can last for years, while other conditions can occur simultaneously. From the perspective of causality, the connections can be divided into two situations: comorbidity and multimorbidity. The former refers to the combined effects of additional conditions in reference to an index chronic condition, and the latter depicts that no single condition holds priority over any of the cooccurring conditions [1]. Sometimes, it is complicated and challenging to sort out this causal relationship and distinguish comorbidities from multimorbidities. But one thing is for sure. For individual patients, multimorbidities or comorbidities are always associated with a greater demand for professional help, a poorer prognosis, greater interference with everyday life, and lower socioeconomic status [2]. Also, higher prevalence, mortality, and disability rate that result from multiple coexisting conditions lead to increased social burdens. Hence, it is imperative to develop a thorough understanding of the association between diseases in individuals.

Can we identify a disorder that puts someone at more risk of developing a second disorder? Increased scientific interest in the underlying relationship between different conditions has led to the generation of many theories and reports. Morikawa et al. revealed the coexistence of adenomyomatosis and primary gallbladder carcinoma [3]. Akpinar pointed out that thyroid dysfunction was an underestimated comorbidity of chronic obstructive pulmonary disease and reviewed the mechanism of the occurrence and the clinical outcome [4]. Wicklein and Gosch reported multimorbidity interactions of osteoporosis with shared pathophysiological mechanisms in older age [5]. Di Angelantonio et al. evaluated the mortality risk and estimated reductions in life expectancy associated with cardiometabolic multimorbidity [6]. In addition, several case reports were published to describe individual patients with concomitant diseases from the same or different body systems such as genitourinary system, digestive system, and circulatory system. [7–9] Although considerable progress towards furthering our understanding of the connections between diseases has been made, most studies had relatively insufficient sample sizes (e.g., case reports), resulting in low epidemiological and statistical significance. Furthermore, almost all researches merely focused on comorbidities or multimorbidities of one disease or one body system. A whole network association remained under investigation.

The association rule mining technique is one of the most popular and effective unsupervised data mining approaches that are always conducted to extract useful information from large amounts of stored data in databases. It is usually applied to discover relations between items in big data [10]. Association rule mining has been used in various medical applications such as detecting near-crash events of traffic accidents [11], mining risk factors of diseases [12], and classifying the care needs of patients [13]. Recently, pattern mining technique was applied on the novel coronavirus (COVID-19) genome sequences to discover frequently occurring nucleotides, sequential relationships between nucleotides, and predict the next nucleotides bases of a sequence [14]. Additionally, running the mining algorithm could help make the medication combination recommendations for obstetric hypertension patients [15]. Apriori algorithm is a classic and great candidate of all association rule mining approaches. It processes by identifying noticeable rules among frequent patterns that are mined first through establishing threshold values of support and confidence [16]. Apriori algorithm-based association rule analysis provides interpretable and intuitive results to inform general trends in the database [17]. It has already been introduced in the field of exploring the comorbidity of attention-deficit hyperactivity disorder for the most critical parameter, “confidence” in the Apriori algorithm, which is arithmetically equal to the “comorbidity” in epidemiology [18, 19].

In this study, we designed a data mining model aiming at discovering frequent rules of associations between diseases that cooccurred in the same individuals by using the Apriori algorithm and the massive electronic medical record (EMR) database of the affiliated hospital of Xuzhou Medical University. We expected that considering and utilizing these associations between disorders would not only provide evidence and clues for further clinical mechanism researches but also prove that the Apriori algorithm was a practical approach for data mining in the EMR database.

## 2. Materials and Methods

### 2.1. Data Sources and Selection Criteria

The raw data in this study were extracted from the electronic medical record database of the affiliated hospital of Xuzhou Medical University, a well-known Tertiary-Class-A medical center in Jiangsu Province, China. Patients from 142 cities and 32 provinces aged from newborn to 115 years old came to the hospital for diagnosis and treatment. The EMR database was established in 2011 and accumulated over 1.53 million records by the end of 2020. So it could be approximated as a population-based database.

Each record in the database contained various sociodemographic and clinical information. Characteristics relevant to this analysis included patients' sex, age, medical record identification number, citizen ID number, and all discharge diagnosis information consisting of codes and corresponding descriptions during the hospitalization. Patients' sex and age at first admission were screened out to estimate the population distribution only, and they would not be involved in the mining model. Many patients had multiple visits to our hospital, and it became the basis of this research. The medical record identification number was used to represent and distinguish each hospitalization. In other words, each hospitalization could generate a medical record identification number, and the medical record system did not consider whether it was the same patient or not. However, the citizen ID number was a different story, and it played an essential role in the constructing of the dataset in the analysis. It was extracted as the personal identifier that allowed for linkage of multiple hospitalizations for the same person. That is to say, different medical records for different hospitalizations of the same person contained the same citizen ID number. Both medical record identification numbers and citizen ID numbers were processed through recoding and original identity erasure to avoid disclosure of the identity of the enrollee. As a result, this study was deemed exempt by the Ethical Committee of the affiliated hospital of Xuzhou Medical University, for we only constituted an analysis of deidentified hospital discharge data within the database, and no human experiment was involved.

Discharge diagnosis information was the critical data of this analysis and served as final diagnosis encoded in the form of codes and descriptions that were listed in International Classification of Diseases, 10th revision (ICD-10) in the database. ICD-10 coding system has been widely used for counting of diseases, injuries, symptoms for epidemiology, prevention, managing health care and allocation of resources for many years. ICD-10 codes are structured by an alphabetical character followed by two digits at the three-character level, then a point and a fourth character. Each character within each position has a specific meaning, allowing for flexibility in expansion and consistency within the coding system. The first alphabetical character usually represents “chapters” that are divided by body system, disease state, or reason for encounter. Then, “chapters” are divided into “categories” represented by three-character codes, and these, in turn, may be subdivided into “subcategories” with specific fourth characters. Although subcategories enable the coding of a disease or condition more specifically, the three-character category codes are always used for international reporting and comparisons and have more epidemiological and statistical characteristics. Hence, for each hospitalization, we scanned all available diagnosis codes that indicated both main conditions and other conditions. Then, we intercepted the first three characters of the full-length code, which was the categories, and incorporated them into the mining model. Furthermore, diagnosis codes from the chapters of “factors influencing health status and contact with health services” (ICD-10 “Z” codes) and “external causes of morbidity and mortality” (ICD-10 “V”, “W”, “X”, and “Y” codes) were excluded for they did not represent any diseases or conditions. Those codes with corresponding descriptions, including the word “other”, were also excluded because the conditions these codes represent could not be simply classified into one category. It was ensured that these codes would not disturb the performance of the model.

Professional coders constructed the code by translating and “abstracting” information from medical documentation written by clinicians and selecting the appropriate value for each of the characters. The coding staff were all well-trained and very familiar with the ICD-10 language, coding structure, and rules. To ensure that everyone who coded with ICD-10 did so in the same way and that the resulting codes were consistent and comparable, the search tools in the EMR system helped coders to easily choose a correct code and clinicians, and coders worked together to ensure the best outcome in terms of the codes assigned. Besides, a rigorous coding protocol was followed. First, two coders independently coded the same cases with preferably a third person to be adjudicator should the two coders disagree. Second, where documentation appeared incomplete or the coder required clarification, advice from the clinicians involved in the case should be sought before a final decision on the appropriate codes for a case was made. Third, if the classification provided a four-character subcategory, then this should be utilized rather than using the higher level three-character category. That is, the assigned codes should be valid, preferably to the lowest level of the classification, to maximize the information that could be extracted from the coded data.

Some records were excluded in this research: (1) patients with single hospitalization during the period (2) diagnosis information containing ICD-10 “V”, “W”, “X”, “Y', and “Z” codes or codes with corresponding descriptions including the word “other” (3) records with incomplete data or missing values.

Considering the coding quality and data integrity, records from Jan 1, 2015, to Dec 31, 2020, were enrolled in this analysis. Finally, 144207 patients with 555565 hospitalizations were selected, and all their diagnosis codes (1551732 codes) and corresponding descriptions consisting of main conditions and other conditions were collected after the data preprocessing and filtering according to the selection criteria.

### 2.2. Data Analysis

Frequent rules of associations between coexisting diseases were mined using the Apriori algorithm. The Apriori algorithm was first presented by R. Agrawal to mine rules in a customer transaction database in 1993 [20] and has been proven to be one of the ten classic algorithms in the field of data mining [12]. Before applying the Apriori algorithm, the extracted data from the EMR were prepared through the data preprocessing step. First, raw data were transformed using the recoded personal identifier to merge the diagnosis information from different hospitalizations of the same individual patient and reconstruct these codes in the same row. The merged dataset represented the match between the patient arrivals and corresponding diagnosis codes that were expressed as “categories” in ICD-10. Second, the notations for each diagnosis code were “True” or “False”. For each transaction, diagnosis codes of the conditions that the patients ever had were represented as “True”, while the other codes were defined as “False” using binary values. The structured dataset that had binary representation was finally prepared for the Apriori algorithm. A sample of the structured dataset is illustrated in Table 1.

A whole collection of the diagnosis codes represented by the binary values in the same row was denoted as a “transaction” which originated in the field of shopping. In one transaction, every diagnosis that the patient ever had was an “item,” and every possible combination of items in the transaction was called “itemset.” So an itemset could contain 1 item, 2 items, or more. Every itemset was a subset of codes from A00 to U99. The purpose of the Apriori algorithm was to extract association rules of each itemset from every transaction. For example, a rule “itemset1 − >itemset2” depicted that the appearance of itemset1 implied the appearance of itemset2 in the same transaction. In this rule, itemset1 and itemset2 were called “antecedent” and “consequent,” respectively. However, it was crucial to note that the implication was just cooccurrence and not traditional deterministic causality. Rules that the Apriori algorithm generated did not have to imply cause and effect necessarily.

A lot of combinations of rules can be mined from the structured dataset once the Apriori algorithm starts. Luckily, not every one of them is meaningful and remarkable. Three kernel values are involved for evaluating the performance of the algorithm and filtering out meaningful rules preliminarily before the manual screening: support, confidence, and lift. The support of itemset1 − >itemset2 is defined as the percentage of transactions in the whole dataset that contains both itemset1 and itemset2 (Equation (1)). In the context of epidemiology, the support of itemset1 − >itemset2 is equivalent to the prevalence rate of both itemset1 and itemset2:

(1) $$\begin{array}{c} \text{Support}\left(\text{itemset}1⟶\text{itemset}2\right)=P\left(\text{itemset}1\cap \text{itemset}2\right). \end{array}$$

“Confidence” is the critical metric in the Apriori algorithm. The confidence of itemset1 − >itemset2 is the conditional probability of occurrence of itemset2, given itemset1 (Equation (2)). In other words, it means the percentage of transactions containing both itemset1 and itemset2 in all transactions containing itemset1. It resembles the comorbidity of itemset2 with itemset1 within the same period in terms of epidemiology:

(2) $$\begin{array}{c} \text{Confidence}\left(\text{itemset}1⟶\text{itemset}2\right)=\frac{P\left(\text{itemset}1\cap \text{itemset}2\right)}{P\left(\text{itemset}1\right)}. \end{array}$$

The lift of itemset1 - > itemset2 is the ratio of the joint probability of itemset1 and itemset2 and product of their marginal probabilities, mathematically (Equation (3)). In sample terms, ‘lift' measures the independence between itemset1 and itemset2. The lift value of an association rule greater than 1 indicates the antecedent itemset and the consequent itemset are dependent and correlated positively. Otherwise, the two itemsets are independent and there's a weak association between them:

(3) $$\begin{array}{c} \text{Lift}\left(\text{itemset}1,\text{itemset}2\right)=\frac{P\left(\text{itemset}1\cap \text{itemset}2\right)}{P\left(\text{itemset}1\right)\text{P}\left(\text{itemset}2\right)}. \end{array}$$

In general, the Apriori algorithm can be simplified in two steps: First, find out all of the frequent sets that are satisfied with a minimum support degree or minimum confidence degree. Second, from these frequent itemsets, strong association rules that meet minimum support and minimum confidence are generated. To avoid generating misleading rules, threshold settings for support, confidence and lift are critical. But there is no universal approach to set up threshold values according to the previous researches. The process of thresholds setting may suffer a certain level of subjectivity, and there is a trade-off between higher or lower support values. Setting a higher threshold value would reduce the number of rules that might result in missing some essential rules with low frequencies and setting a lower threshold value could result in a large number of rules that might hinder the management from summarizing rules because too many rules should be examined and interpreted manually. Besides, a high lift value suggests the strong dependency between the antecedent and consequent, and an association rule containing the two itemsets would be worthy of reporting if the lift value of this rule is high. This is an advantage of the Apriori algorithm to discover some less frequent but important patterns. Thus, many rounds of testing and evaluation were done before defining final thresholds to mine reasonable rules and to ensure the robustness of the model performance. Considering the vast amounts of types of diseases in the dataset, the rules satisfying support ≥ 0.001, confidence ≥ 60%, and lift > 1 were selected. Rules were sorted by confidence in descending order because the ones with the highest confidence value were the ones most interesting. After being filtered with thresholds, all the extracted rules were validated and reviewed by experts to remove duplicates and intermediate items and to ensure they were in line with basic scientific facts. Finally, rules with antecedent containing no more than two items (two ICD-10 diagnosis code categories) and consequent containing only one item (one ICD-10 diagnosis code category) were chosen for too many items in antecedent or consequent would result in relatively low population representation.

In this study, data query and extraction were conducted in the EMR database that was constructed based on ORACLE 10 g (Integrated Development Environment: PL/SQL Developer 7.1.5.1399). Data preprocessing and the Apriori algorithm were employed by the package “pandas” (ver.1.1.5) and “mlxtend” (ver.0.18.0) in Python 3.6.4 (Anaconda3 ver.5.1.0), respectively. Visualization of the result was fitted using Excel 2016.

The data extracted from the EMR database was stored in “Comma-Separated values” (.csv) format before applying the algorithm. The data file consumed approximately 70 MB, which was not actually regarded as large-scale data compared to the real big data file. However, the Apriori algorithm has a common drawback when handling data: it processes slowly because it considers the whole transaction database. In order to address this issue, we imported the package “joblib” (ver.0.13.2) to implement parallel computation in Python using a quad-core CPU. The execution time was shortened to nearly a quarter of the original time when just using the single thread of CPU.

## 3. Results

### 3.1. Descriptive Characteristics of the Participants and the Corresponding Extracted Diagnosis Information

Among 144207 participants in this study, 73133 male patients' diagnosis information was extracted, while the female cases were 71074. The median age of all participants at first admission was 56 years old, and the minimum age, lower-quartile age, upper-quartile age, and maximum age were 1d, 42 years old, 67 years old, and 102 years old, respectively. The age distribution is represented in Figure 1. All enrollees were hospitalized at least two times and the highest frequency of hospitalizations in one individual was 102.

1551732 codes from these participants' diagnosis information were intercepted and classified into 1268 ICD-10 categories that accounted for 79.7% of all ICD-10 categories (1591 categories except for “V”, “W”, “X”, “Y”, and “Z” code). The frequency distributions of diagnosis codes classified by “chapters” (first alphabetical character) and “categories” (first three characters) are shown in Figures 2 and 3, respectively. When classified by “chapters”, the most prevalent disease cluster was “disease of the circulatory system” (“I” codes, 28.60%), followed by “neoplasms” (“C” codes, 20.13%), “endocrine, nutritional and metabolic diseases” (“E” codes, 9.20%), “diseases of the digestive system” (“K” codes, 7.65%), “diseases of the respiratory system” (“J” codes, 6.62%). When classified by “categories”, the most prevalent disease cluster was “essential (primary) hypertension” (“I10” code, 9.62%), followed by “cerebral infarction” (“I63” code, 6.19%), “type 2 diabetes mellitus” (“E11” code, 5.47%), “chronic ischaemic heart disease” (“I25” code, 3.58%), “malignant neoplasm of bronchus and lung” (“C34” code, 3.53%), “malignant neoplasm of breast” (“C50” code, 3.18%), “pneumonia, organism unspecified” (“J18” code, 1.68%), “gastritis and duodenitis” (“K29” code, 1.61%), “angina pectoris” (“I20” code, 1.59%), and “chronic kidney disease” (“N18” code, 1.28%). Among the 1268 ICD-10 categories, five categories reached the frequency level of more than 50000. Twenty-two categories reached the frequency level of 10000-49999. One hundred eighty-eight categories reached the frequency level of 1000-9999. Four hundred fourteen categories reached the frequency level of 100-999. Six hundred thirty-nine categories reached the frequency level of 1-99.

To avoid missing any critical association rule, we set the support threshold to 0.001 at the beginning, and no minimum confidence or lift thresholds were limited. 12889 rules were generated after running the Apriori algorithm on the preprocessed dataset. One hundred ten rules were finally kept through threshold filtering and manual examination. In order to clarify associations between diseases, we divided these mined rules into two parts according to ICD-10 “chapters” that usually represented body systems: associations between different ICD-10 “chapters” and associations within the same ICD-10 “chapter.”

### 3.2. Association Rule Mining between Different ICD-10 “Chapters”

Among 110 rules, there were 13 rules whose antecedent codes and consequent codes came from different ICD-10 “chapters” (Table 2). All consequents of the rules were about the diseases of the circulatory system—essential (primary) hypertension and cerebral infarction. Type 2 diabetes mellitus (E11) appeared most—in five rules as antecedents, and it seemed to have a strong relationship with essential hypertension and cerebral infarction. These rules were ordered by confidence degree from largest to smallest. The highest association was the rule “chronic kidney disease (N18) and type 2 diabetes mellitus (E11) -> essential (primary) hypertension (I10)” with confidence of 83.61% that meant the ratio of the cooccurrence rate of chronic kidney disease, type 2 diabetes mellitus, and hypertension over the prevalence of chronic kidney disease combined with type 2 diabetes mellitus. The support value of 1.08% indicated the prevalence of the three diseases within a certain period. The lift value of 1.98 suggested that chronic kidney disease combined with type 2 diabetes mellitus is positively associated with essential hypertension. The second rule “Parkinson's disease (G20) -> cerebral infarction (I63)” showed that individuals who have Parkinson's disease are most likely to experience cerebral infarction (83.55% probability). The third rule, “transient cerebral ischaemic attacks and related syndromes (G45) and type 2 diabetes mellitus (E11) -> cerebral infarction (I63)” depicted that the group with the second largest probability of experiencing cerebral infarction (83.18%) is those who have transient cerebral ischaemic attacks and related syndromes and type 2 diabetes mellitus. Rule 5 indicated that patients with hemiplegia have the highest probability of encountering essential hypertension in those rules whose antecedents contain just one item.

One crucial result which needed to be highlighted was that patients who have chronic kidney disease combined with type 2 diabetes mellitus have more risks to experience essential hypertension than those who only suffer from one of the two diseases according to rule 1, rule 6, and rule 12. Besides, if both transient cerebral ischaemic attacks and type 2 diabetes mellitus rather than only the former one were observed in a patient, it was highly probable for this patient to acquire cerebral infarction on the basis of rule 3 and rule 4. In addition, spinal disease and hypothyroidism were associated with cerebral infarction based on rule 8, rule 9, and rule 13, which might be an innovative discovery.

### 3.3. Association Rule Mining within the Same ICD-10 “Chapter”

Ninety-seven rules were selected while considering those whose antecedent codes and consequent codes were from the same “chapter” (Table 3). 26 ICD-10 categories from 12 “chapters” were involved from the perspective of the consequent codes. There were 55 rules (56.70%) whose consequent codes represented diseases of the circulatory system, followed by 12 rules (diseases of the digestive system, 12.37%) and 9 rules (diseases of the respiratory system, 9.28%). The rest rules were distributed in the fields of “neoplasms” (4 rules), “injury, poisoning and certain other consequences of external causes” (3 rules), “diseases of the eye and adnexa” (3 rules), “endocrine, nutritional and metabolic diseases” (2 rules), “congenital malformations, deformations and chromosomal abnormalities” (2 rules), “symptoms, signs and abnormal clinical and laboratory findings, not elsewhere classified” (2 rules), “mental and behavioral disorders” (2 rules), “diseases of the nervous system” (2 rules), and “certain infectious and parasitic diseases” (1 rule). There were eight rules (8.25% of 97 rules) whose confidence degree was greater than 90%. Twenty-six rules' confidence degree was between 80% and 90% (accounting for 26.80%). 50 rules' confidence degree was between 70% and 80% (51.55%). 13 rules' confidence degree was between 60% and 70% (13.40%). The highest confidence degree was achieved in the rule “congenital malformations of gallbladder, bile ducts and liver (Q44) -> cystic kidney disease (Q61)” whose confidence degree was 97.27%. The highest support degree was found in two rules: “cerebral infarction (I63) -> essential (primary) hypertension (I10)” and “essential (primary) hypertension (I10) -> cerebral infarction (I63),” whose support value was 48.68%. Rule “Malignant neoplasm of renal pelvis (C65) -> Malignant neoplasm of kidney, except renal pelvis (C64)” achieved the highest lift degree (27.80), which meant malignant neoplasm of the renal pelvis and other malignant neoplasms of the kidney were highly dependent.

Some worth emphasizing results were discovered when we took a panoramic view: (1) Rule 61 “acute myocardial infarction -> chronic ischaemic heart disease” suggested an acute attack from a chronic disease. (2) Some rules indicated the spreading of a disease from an original site to one or more sites elsewhere in the body, e.g., cancer metastasis, based on rule 7, rule 13, rule 45, rule 82, and rule 83. (3) The exacerbation of diseases could be seen in rule 4, rule 6, rule 86, and rule 90. (4) Patients who have two combined conditions in antecedent usually have more risks to experience the specific disease in consequent than those who only suffer from one of the two diseases in antecedent, which was consistent with the above conclusion. (5) “Congenital malformations of gallbladder, bile ducts and liver” (Q44) and “cystic kidney disease” (Q61) were associated with each other according to rule 1 and rule 3.

“Essential (primary) hypertension” (I10) appeared most frequently as the consequent of rules (40 rules), followed by “cerebral infarction” (I63, 11 rules) and “pneumonia, organism unspecified” (J18, 9 rules). Common circulatory system diseases, like essential hypertension, cerebral infarction, atherosclerosis, intracerebral haemorrhage, chronic ischaemic heart disease, and angina pectoris, are mutual inducing factors. When patients experience more circulatory system diseases, they are at increased risk for other disorders in the circulatory system. Among 40 rules about essential hypertension, the rule with the highest confidence was the rule “atherosclerosis (I70) and intracerebral haemorrhage (I61) -> essential hypertension (I10)” with confidence: 89.04%. There were seven rules whose antecedent contained a single ICD-10 category in the 40 rules. Among them, the rule with only intracerebral haemorrhage as antecedent obtained the highest confidence degree: 82.09%. “Occlusion and stenosis of precerebral arteries, not resulting in cerebral infarction” (I66) and “sequelae of cerebrovascular disease” (I69) were the most frequent items in antecedents of the rules about hypertension. Each of them appeared in 10 rules. Eleven rules described the relationship between other diseases and cerebral infarction, and the rule with the highest confidence was the rule “occlusion and stenosis of cerebral arteries, not resulting in cerebral infarction (I66) -> cerebral infarction (I63)” with confidence: 96.05%. “Atherosclerosis” (I70) appeared most frequently in the antecedents of the rules about cerebral infarction (5 rules), which indicated that patients with atherosclerosis have a relatively higher probability of suffering from cerebral infarction. Finally, when considering rules whose consequent was pneumonia (J18), acute respiratory conditions like tonsillitis, bronchiolitis, laryngitis, and tracheitis, all had the potential to develop into pneumonia. Rule “acute tonsillitis (J03) combined with acute laryngitis and tracheitis (J04) -> pneumonia, organism unspecified (J18)” achieved the highest confidence degree of all rules concerning pneumonia: 82.22%. The rule with only acute bronchiolitis as antecedent obtained the highest confidence degree: 80.80% in 4 rules whose antecedent contained a single item. “Acute tonsillitis” (J03) was the most frequent item that appeared in the antecedent position of rules about pneumonia (5 rules).

## 4. Discussion

Data mining is a fantastic technology that combines machine learning, statistics, big data technology, and artificial intelligence. It consists of classification, association analysis, outlier detection, clustering, and forecasting. These functions have already been conducted in many medical researches, especially in classifying patients [21] and generating predictions [22]. However, to the best of the knowledge, the use of association analysis is rare in the context of multimorbidity relationship mining, especially the whole network association. Thus, this study might be the first research which was intended to make a relatively comprehensive understanding of the network associations between different diseases from nearly all body systems by data mining technique using real-life data received from a large-scale diagnosis information database. Recently, deep learning technique, such as deep neural network (DNN), is very famous in the field of data mining. It has outperformed the conventional data mining techniques in identifying complex patterns. However, this comes at an expensive cost: opaqueness and uninterpretability. The “black-box” is difficult to debug and isolate the reason behind certain outcomes because deep learning algorithms lack strong theoretical backing [23]. The Apriori algorithm contrasts this situation, for it is very simple to explain and has a solid theoretical basis. Consequently, the Apriori algorithm became our choice in this research.

As shown above, association rules about the circulatory system and metabolic diseases accounted for a major part of the results. One of the principal explanations for this phenomenon is that the operating mechanism of the Apriori algorithm forces the number of the item to occupy a certain proportion in the dataset before the rules of the item can be displayed. In other words, if the rule about a particular disease wants to be selected, the support degree of this disease needs to reach a given level. In recent years, circulatory system disease has contributed more and more to the increase of the morbidity and prevalence in the disease spectrum of China. Rao et al. [24] conducted an epidemiologic survey in China and estimated the prevalence of circulatory system diseases in 2013 and 2018. The prevalence rate increased substantially from 14.25% to 21.25%. When sorted by prevalence, the top three circulatory system disease was hypertension (17.81%), cerebrovascular disease (1.65%), and angina pectoris (0.08%). The result from this epidemiologic research was basically consistent with the percentage of circulatory system disease in our dataset. Also, it proved that the database used in this study was approximately population-based. Hence, what we mined was not surprising.

As a kind of chronic underlying disease cluster, there is no complete cure for cardiovascular and cerebrovascular diseases at present. Many patients live with, rather than die from, these chronic health conditions. Cardiovascular and cerebrovascular diseases devastate patients' bodies and minds for a long time, resulting in poor physical fitness. Most patients survive long enough to suffer the long-term consequences and are very prone to other conditions during the period, which can also be seen as a potential connection with other diseases. One circulatory system disease always induces one or more other circulatory disorders in an individual. In addition, the more circulatory system diseases occur in one individual, the more likely the patient is to suffer from another circulatory system disease. Thiene and Valente [25] reported that hypertension is usually associated with aortic dissecting aneurysm, and angina pectoris and myocardial infarction are the complications of coronary atherosclerosis that is the primary cause of death in the elderly. Roberts [26] found that hypertension appears to be a common and underlying risk factor to developing various cardiovascular conditions, like cerebral arterial rupture, hyperlipidemia, and atherosclerosis. Liu et al. [27] analyzed the characteristics and clinical medicine information of 4497 patients with Parkinson's syndrome in 17 hospitals all over China from diagnostic information databases of hospital information systems. The results indicated the most common comorbidities of Parkinson's syndrome are cerebral infarction, hypertension, coronary heart disease, diabetes, and lung infections. The combined incidence of hypertension reached 33.46%. Besides the epidemiologic data, the pathological mechanism of comorbidities or multimorbidities in cardiovascular diseases has been depicted by scholars. High serum urate levels are influenced by genetic pleiotropy, which could be considered a common cause resulting in an increased risk of different types of cardiac events [28]. Multiple drugs, including long-chain polyunsaturated fatty acids [29] and cannabidiol [30], have been proven effective in treating Parkinson's syndrome, ischaemic stroke, cerebral infarction, hypertension, and diabetes, which indicates that these disorders may have similar pathogenic sites and principles. In addition to the mutual induction between circulatory system diseases, cardiovascular and cerebrovascular diseases are also related to the disorders from other body systems. Hypothyroidism, spondylosis, cervical spine injury, and chronic kidney disease are all reported to be directly or indirectly associated with circulatory system diseases [31–35]. In general, the above researches presented a connection network about circulatory system diseases, which was consistent with our findings.

Lower support values were found in those association rules about disorders from other body systems, for the number of the total samples was very large, and the prevalence of these diseases was relatively lower compared with circulatory system diseases. It did not mean that the association degree between these conditions was weak or these rules were not important. On the contrary, these rules were very applicable to predict the occurrence and development of diseases from other body systems except circulatory system disorders. As described above, pneumonia could become a concomitant condition and terminal stage of acute respiratory illnesses, like tonsillitis and bronchiolitis [36, 37]. Congenital malformations of the gallbladder, bile ducts, and liver are always accompanied by polycystic kidney disease [38, 39]. Malignant neoplasm of renal pelvis tends to metastasize to surrounding area parts of the kidney (e.g., adrenal gland) [40, 41]. These works of literature prove that the association rules that we mined are valid and in line with clinical practice.

The aim of this study was not only to provide the necessary evidence for known connections between disorders but also to generate predictive relationship patterns. Some rules were temporarily not reported by existing clinical or epidemiologic researches, and they have not been fully discovered or valued. In these rules, there was no obvious or easy-to-detect clinical link between diseases. But the disorders might share common risk factors, or they themselves were intermediate states of other conditions. These rules could be regarded as the beginning and clues of mechanism researches on the associations.

## 5. Limitations and Future Perspectives

Our research has several limitations. First, it is believed that connections between many diseases can be maintained for decades. Limited by objective circumstances, such as data quality and database access authorization, only 6-years' hospitalization and diagnosis information in a unique hospital was calculated instead of the whole lifetime samples, which might lead to the omission of some long-lasting association information. If possible, a multicenter study can help validate the generated rules and more exciting results will be discovered. Second, the occurrence of diseases can be influenced by many psychosocial factors. However, we did not measure these factors, and they were not incorporated into the model in this analysis because the dataset anonymized participants to avoid possible misuse. Besides, the Apriori algorithm is a big data screening approach, and it is not designed to present or analyze those detailed information, which limits our conclusion in this respect. Further in-depth subgroup analysis should be conducted by using advanced techniques. Last but not least, we could not reach conclusions regarding the causality due to the characteristics and disadvantages of the Apriori algorithm. All the connections reported above could only be considered a correlation, but it does not prevent the mined rules from becoming clues to further clinical researches.

As mentioned above, the main limitation of the traditional association rule mining algorithms is the database format where only binary items can be mined. The antecedent and the consequent are not traditional deterministic causality. To address this issue, we plan to implement the sequential pattern mining (SPM) technique in further research. SPM is an extension of association rule mining to discover a set of ordered patterns in a sequence database. It is designed to discover and analyze statistically relevant subsequences from items with time constraints [42]. Consequently, it is more suitable to detect the chronological order and causal relationship of disease occurrence. Furthermore, a multicenter study with longer test period implies huge memory cost, low processing speed, and inadequate hard disk space. Several newly developed distributed data mining frameworks, including Decomposition Transaction for Distributed Pattern Mining (DT-DPM) [43], Cluster-based Retrieval using Pattern Mining (CRPM) [44], and Clustering-Based Pattern Mining (CBPM) [45, 46], may aid in boosting the performance by partitioning the whole database using a clustering algorithm, then computing the local results, and merging the results eventually. In addition, high-performance computing is based on exploiting the massively threaded computing of Graphics Processing Units (GPU) to conduct a parallel mining process. These advanced frameworks may be applied in our future research.

## 6. Conclusion

Connections about different diseases have not been fully acknowledged until now. This study elucidated the interesting network associations between disorders from different body systems and demonstrated the usefulness of the Apriori algorithm in comorbidity or multimorbidity study in a large-scale EMR database. Cooccurrence of diseases may worsen each other's prognosis, reduce the efficacy of treatments, and increase mortality. In addition, the family and social burden of comorbidity and multimorbidity remain a major issue. Doctors, scholars, policy-makers, or even patients should address this growing challenge by renewing recognition. In this analysis, disorders from the mined association rules could become the indicators of other conditions, which led to improved prevention strategies and the early identification of patients at risk. Monitoring related diseases based on these predictive patterns is also useful to aid in assessing the quality of life, clinical treatment decision-making, and minimizing the coexisting disorders' impact on the mortality eventually. Finally, the Apriori algorithm still needs further dynamic evidence for establishing causal relationships. Future clinical researches are required and should concentrate on verifying these mined connections.

## Figures and Tables

**Figure 1:** Frequency distribution of age.

**Figure 2:** Frequency distribution of diagnosis codes classified by ICD-10 “chapters” (first alphabetical character).

**Figure 3:** Partial frequency distribution of diagnosis codes classified by ICD-10 “categories” (first three characters) (top 30).

**Table 1:** Sample of structured dataset.

Personal Identifier	A00	A01	A02	…	A99	B01	B02	…	B99	C01	C02	C03	…	C97	…	T01	T02	…	T98	…	U85
*P* i	FALSE	FALSE	TRUE	FALSE	FALSE	FALSE	FALSE	TRUE	FALSE	FALSE	FALSE	FALSE	FALSE	TRUE	FALSE	FALSE	FALSE	FALSE	FALSE	FALSE	FALSE
*P* i + 1	FALSE	FALSE	FALSE	TRUE	FALSE	FALSE	FALSE	FALSE	FALSE	FALSE	FALSE	TRUE	FALSE	FALSE	FALSE	FALSE	FALSE	FALSE	FALSE	FALSE	FALSE
*P* i + 2	FALSE	FALSE	FALSE	FALSE	FALSE	TRUE	FALSE	FALSE	FALSE	FALSE	FALSE	TRUE	FALSE	FALSE	FALSE	TRUE	FALSE	FALSE	FALSE	TRUE	FALSE
*P* i + 3	TRUE	FALSE	FALSE	FALSE	FALSE	FALSE	FALSE	FALSE	TRUE	TRUE	FALSE	FALSE	FALSE	FALSE	TRUE	FALSE	FALSE	FALSE	FALSE	FALSE	FALSE
*P* i + 4	FALSE	FALSE	TRUE	FALSE	FALSE	FALSE	FALSE	TRUE	FALSE	FALSE	FALSE	FALSE	FALSE	FALSE	FALSE	FALSE	FALSE	FALSE	FALSE	FALSE	FALSE
*P* i + 5	FALSE	FALSE	TRUE	FALSE	FALSE	FALSE	FALSE	FALSE	FALSE	FALSE	FALSE	FALSE	FALSE	FALSE	TRUE	FALSE	FALSE	FALSE	FALSE	FALSE	FALSE
*P* i + 6	FALSE	FALSE	FALSE	FALSE	FALSE	TRUE	TRUE	FALSE	FALSE	FALSE	TRUE	TRUE	FALSE	FALSE	FALSE	FALSE	FALSE	FALSE	FALSE	FALSE	FALSE
*P* i + 7	FALSE	FALSE	FALSE	FALSE	TRUE	FALSE	FALSE	FALSE	FALSE	FALSE	FALSE	FALSE	FALSE	FALSE	FALSE	FALSE	FALSE	FALSE	FALSE	TRUE	FALSE
*P* i + 8	FALSE	TRUE	FALSE	FALSE	FALSE	FALSE	FALSE	FALSE	FALSE	FALSE	FALSE	FALSE	FALSE	FALSE	FALSE	FALSE	TRUE	FALSE	TRUE	FALSE	FALSE
*P* i + 9	FALSE	FALSE	FALSE	FALSE	FALSE	FALSE	FALSE	FALSE	FALSE	TRUE	FALSE	FALSE	FALSE	FALSE	FALSE	FALSE	FALSE	TRUE	FALSE	FALSE	FALSE
*P* i + 10	FALSE	FALSE	FALSE	FALSE	FALSE	FALSE	FALSE	FALSE	FALSE	FALSE	TRUE	TRUE	FALSE	FALSE	FALSE	FALSE	FALSE	FALSE	FALSE	FALSE	FALSE

**Table 2:** Association rules between different ICD-10 “chapters”.

No.	Association rules (ICD-10 codes)	Antecedent	Consequent	Support	Confidence	Lift
1	N18, E11 - > I10	Chronic kidney disease type 2 diabetes mellitus	Essential (primary) hypertension	1.08%	83.61%	1.98
2	G20 - > I63	Parkinson's disease	Cerebral infarction	1.01%	83.55%	2.16
3	G45, E11 - > I63	Transient cerebral ischaemic attacks and related syndromes type 2 diabetes mellitus	Cerebral infarction	1.05%	83.18%	2.15
4	G45 - > I63	Transient cerebral ischaemic attacks and related syndromes	Cerebral infarction	3.80%	78.97%	2.17
5	G81 - > I10	Hemiplegia	Essential (primary) hypertension	1.08%	73.21%	1.77
6	N18 - > I10	Chronic kidney disease	Essential (primary) hypertension	2.90%	70.28%	1.81
7	G45, E11 - > I10	Transient cerebral ischaemic attacks and related syndromes type 2 diabetes mellitus	Essential (primary) hypertension	1.05%	70.22%	1.35
8	M50 - > I63	Cervical disc disorders	Cerebral infarction	1.74%	68.27%	1.91
9	M47 - > I63	Spondylosis	Cerebral infarction	2.15%	66.25%	1.85
10	E14 - > I10	Unspecified diabetes mellitus	Essential (primary) hypertension	2.04%	62.74%	1.61
11	J18, E11 - > I63	Pneumonia, organism unspecified type 2 diabetes mellitus	Cerebral infarction	1.01%	62.13%	1.57
12	E11 - > I10	Type 2 diabetes mellitus	Essential (primary) hypertension	11.73%	61.49%	1.58
13	E02 - > I63	Subclinical iodine-deficiency hypothyroidism	Cerebral infarction	1.02%	60.79%	1.49

**Table 3:** Association rules within the same ICD-10 “chapter”.

No.	Association rules (ICD-10 codes)	Antecedent	Consequent	Support	Confidence	Lift
1	Q44 -> Q61	Congenital malformations of the gallbladder, bile ducts, and liver	Cystic kidney disease	19.89%	97.27%	4.71
2	K80, K20 -> K29	Cholelithiasis and oesophagitis	Gastritis and duodenitis	0.33%	96.77%	1.81
3	Q61 -> Q44	Cystic kidney disease	Congenital malformations of the gallbladder, bile ducts, and liver	19.89%	96.40%	4.71
4	I66 -> I63	Occlusion and stenosis of cerebral arteries, not resulting in cerebral infarction	Cerebral infarction	5.94%	96.05%	1.46
5	I66, I25 -> I63	Occlusion and stenosis of cerebral arteries, not resulting in cerebral infarction chronic ischaemic heart disease	Cerebral infarction	1.73%	94.69%	1.44
6	I65 -> I63	Occlusion and stenosis of precerebral arteries, not resulting in cerebral infarction	Cerebral infarction	5.01%	92.64%	1.41
7	K20 -> K29	Oesophagitis	Gastritis and duodenitis	4.15%	92.25%	1.73
8	R13 -> R47	Dysphagia	Speech disturbances, not elsewhere classified	12.15%	90.91%	5.77
9	I70, I61 -> I10	Atherosclerosis intracerebral haemorrhage	Essential (primary) hypertension	0.13%	89.04%	1.24
10	G80 -> G40	Cerebral palsy	Epilepsy	1.35%	86.54%	3.94
11	I61, I69 -> I10	Intracerebral haemorrhage sequelae of cerebrovascular disease	Essential (primary) hypertension	1.11%	86.32%	1.20
12	I61, I25 -> I10	Intracerebral haemorrhagechronic ischaemic heart disease	Essential (primary) hypertension	0.64%	86.14%	1.20
13	K21 -> K29	Gastroesophageal reflux disease	Gastritis and duodenitis	4.15%	85.71%	1.61
14	I20, I69 -> I10	Angina pectoris sequelae of cerebrovascular disease	Essential (primary) hypertension	0.39%	84.78%	1.18
15	I70, I69 -> I10	Atherosclerosis sequelae of cerebrovascular disease	Essential (primary) hypertension	0.20%	84.48%	1.18
16	I25, I69 -> I10	Chronic ischaemic heart disease sequelae of cerebrovascular disease	Essential (primary) hypertension	1.10%	84.19%	1.17
17	I25, I71 ->I10	Chronic ischaemic heart disease aortic aneurysm and dissection	Essential (primary) hypertension	0.17%	83.84%	1.17
18	I20, I66 -> I10	Angina pectoris occlusion and stenosis of cerebral arteries, not resulting in cerebral infarction	Essential (primary) hypertension	0.54%	83.44%	1.16
19	I80, I61 -> I10	Phlebitis and thrombophlebitis intracerebral haemorrhage	Essential (primary) hypertension	0.12%	83.33%	1.16
20	I20, I61 -> I10	Angina pectoris intracerebral haemorrhage	Essential (primary) hypertension	0.22%	82.71%	1.15
21	I61, I63 -> I10	Intracerebral haemorrhage cerebral infarction	Essential (primary) hypertension	2.20%	82.41%	1.15
22	J03, J04 -> J18	Acute tonsillitis acute laryngitis and tracheitis	Pneumonia, organism unspecified	0.48%	82.22%	1.47
23	I61 -> I10	Intracerebral haemorrhage	Essential (primary) hypertension	3.99%	82.09%	1.15
24	I66, I61 -> I10	Occlusion and stenosis of cerebral arteries, not resulting in cerebral infarction intracerebral haemorrhage	Essential (primary) hypertension	0.21%	82.03%	1.14
25	I50, I65 -> I10	Heart failure occlusion and stenosis of precerebral arteries, not resulting in cerebral infarction	Essential (primary) hypertension	0.21%	81.54%	1.14
26	I71, I63 -> I10	Aortic aneurysm and dissection cerebral infarction	Essential (primary) hypertension	0.24%	81.25%	1.13
27	I70, I10 -> I63	Atherosclerosis essential (primary) hypertension	Cerebral infarction	3.40%	81.08%	1.23
28	I70 -> I63	Atherosclerosis	Cerebral infarction	5.18%	81.05%	1.23
29	I66, I25 -> I10	Occlusion and stenosis of cerebral arteries, not resulting in cerebral infarction chronic ischaemic heart disease	Essential (primary) hypertension	1.48%	80.97%	1.13
30	J21 -> J18	Acute bronchiolitis	Pneumonia, organism unspecified	2.08%	80.80%	1.44
31	K65, K70 ->K74	Peritonitis alcoholic liver disease	Fibrosis and cirrhosis of the liver	0.55%	80.65%	5.85
32	I20, I65 ->I10	Angina pectoris occlusion and stenosis of precerebral arteries, not resulting in cerebral infarction	Essential (primary) hypertension	0.67%	80.43%	1.12
33	I66, I69 -> I10	Occlusion and stenosis of cerebral arteries, not resulting in cerebral infarction sequelae of cerebrovascular disease	Essential (primary) hypertension	0.47%	80.34%	1.12
34	I71 -> I10	Aortic aneurysm and dissection	Essential (primary) hypertension	0.49%	80.00%	1.12
35	I70, I25 -> I63	Atherosclerosis chronic ischaemic heart disease	Cerebral infarction	1.77%	79.53%	1.21
36	I69 -> I10	Sequelae of cerebrovascular disease	Essential (primary) hypertension	4.05%	79.39%	1.11
37	K26 -> K29	Duodenal ulcer	Gastritis and duodenitis	3.91%	79.06%	1.48
38	I65, I69 -> I10	Occlusion and stenosis of precerebral arteries, not resulting in cerebral infarction sequelae of cerebrovascular disease	Essential (primary) hypertension	0.28%	78.77%	1.10
39	I63, I69 -> I10	Cerebral infarction sequelae of cerebrovascular disease	Essential (primary) hypertension	3.04%	78.47%	1.09
40	I25, I65 -> I10	Chronic ischaemic heart disease occlusion and stenosis of precerebral arteries, not resulting in cerebral infarction	Essential (primary) hypertension	1.52%	78.17%	1.09
41	I66, I65 -> I10	Occlusion and stenosis of cerebral arteries, not resulting in cerebral infarction occlusion and stenosis of precerebral arteries, not resulting in cerebral infarction	Essential (primary) hypertension	1.29%	77.95%	1.09
42	J21, J03 -> J18	Acute bronchiolitis acute tonsillitis	Pneumonia, organism unspecified	0.40%	77.50%	1.38
43	H40, H04 ->H25	Glaucoma disorders of lacrimal system	Senile cataract	0.72%	77.42%	2.04
44	I95 -> I63	Hypotension	Cerebral infarction	0.13%	77.38%	1.17
45	C65 -> C64	Malignant neoplasm of the renal pelvis	Malignant neoplasm of the kidney, except the renal pelvis	0.47%	77.19%	27.80
46	R47 -> R13	Speech disturbances, not elsewhere classified	Dysphagia	12.15%	77.18%	5.77
47	J04 -> J18	Acute laryngitis and tracheitis	Pneumonia, organism unspecified	2.14%	76.38%	1.36
48	I70, I50 -> I10	Atherosclerosis heart failure	Essential (primary) hypertension	0.34%	76.15%	1.06
49	I70, I20 -> I63	Atherosclerosis angina pectoris	Cerebral infarction	0.71%	76.14%	1.16
50	I05 -> I48	Rheumatic mitral valve diseases	Artrial fibrillation and flutter	0.43%	75.89%	8.25
51	I70, I20 -> I10	Atherosclerosis angina pectoris	Essential (primary) hypertension	0.70%	75.49%	1.05
52	I70, I66 -> I10	Atherosclerosis occlusion and stenosis of precerebral arteries, not resulting in cerebral infarction	Essential (primary) hypertension	0.45%	75.17%	1.05
53	I20, I63 ->I10	Angina pectoris cerebral infarction	Essential (primary) hypertension	7.95%	75.10%	1.05
54	B91 -> B18	Sequelae of poliomyelitis	Chronic viral hepatitis	0.31%	75.00%	2.19
55	H72 -> H66	Perforation of tympanic membrane	Suppurative and unspecified otitis media	0.72%	75.00%	16.17
56	I48, I66 -> I10	Artrial fibrillation and flutter occlusion and stenosis of precerebral arteries, not resulting in cerebral infarction	Essential (primary) hypertension	0.27%	75.00%	1.05
57	I50, I69 -> I10	Heart failure sequelae of cerebrovascular disease	Essential (primary) hypertension	0.35%	74.89%	1.04
58	J03, J20 -> J18	Acute tonsillitis and acute bronchitis	Pneumonia, organism unspecified	1.93%	74.44%	1.33
59	I66, I50 -> I10	Occlusion and stenosis of precerebral arteries, not resulting in cerebral infarction heart failure	Essential (primary) hypertension	0.19%	74.42%	1.04
60	I66, I63 -> I10	Occlusion and stenosis of precerebral arteries, not resulting in cerebral infarction	Essential (primary) hypertension	4.42%	74.34%	1.04
61	I21 -> I25	Acute myocardial infarction	Chronic ischaemic heart disease	4.70%	74.21%	1.79
62	I66 -> I10	Occlusion and stenosis of precerebral arteries, not resulting in cerebral infarction	Essential (primary) hypertension	4.58%	74.08%	1.03
63	I80, I69 ->I10	Phlebitis and thrombophlebitis sequelae of cerebrovascular disease	Essential (primary) hypertension	0.12%	74.07%	1.03
64	I48, I70 -> I63	Artrial fibrillation and flutter atherosclerosis	Cerebral infarction	0.32%	74.07%	1.12
65	J03 -> J18	Acute tonsillitis	Pneumonia, organism unspecified	9.44%	74.06%	1.32
66	G97 -> G91	Postprocedural disorders of nervous system, not elsewhere classified	Hydrocephalus	1.71%	74.03%	8.32
67	I70, I25 ->I10	Atherosclerosis chronic ischaemic heart disease	Essential (primary) hypertension	1.65%	74.00%	1.03
68	I63 -> I10	Cerebral infarction	Essential (primary) hypertension	48.68%	73.86%	1.03
69	D06 -> D25	Carcinoma in situ of the cervix uteri	Leiomyoma of the uterus	3.04%	73.38%	3.53
70	I00 -> I10	Rheumatic fever without mention of heart involvement	Essential (primary) hypertension	0.12%	73.17%	1.02
71	I65, I63 -> I10	Occlusion and stenosis of precerebral arteries, not resulting in cerebral infarction	Essential (primary) hypertension	3.66%	72.95%	1.02
72	I25, I63 -> I10	Chronic ischaemic heart disease and cerebral infarction	Essential (primary) hypertension	16.95%	72.90%	1.02
73	I65 -> I10	Occlusion and stenosis of precerebral arteries, not resulting in cerebral infarction	Essential (primary) hypertension	3.94%	72.78%	1.02
74	I48, I70 -> I10	Artrial fibrillation and flutter atherosclerosis	Essential (primary) hypertension	0.32%	72.22%	1.01
75	K44 -> K29	Diaphragmatic hernia	Gastritis and duodenitis	1.68%	72.21%	1.35
76	J04, J20 ->J18	Acute laryngitis and tracheitis acute bronchitis	Pneumonia, organism unspecified	0.53%	72.17%	1.29
77	H04 ->H25	Disorders of lacrimal system	Senile cataract	5.09%	71.91%	1.89
78	S93 -> S82	Dislocation, sprain, and strain of joints and ligaments at ankle and foot level	Fracture of the lower leg, including the ankle	1.61%	71.70%	4.85
79	S32, S06 -> S22	Fracture of the lumbar spine and pelvis intracranial injury	Fracture of the rib(s), sternum, and thoracic spine	2.76%	70.65%	2.08
80	E02, E79 -> E11	Subclinical iodine-deficiency hypothyroidism disorders of purine and pyrimidine metabolism	Type 2 diabetes mellitus	0.20%	70.27%	1.04
81	F84 -> F79	Pervasive developmental disorders	Unspecified mental retardation	18.96%	70.18%	2.64
82	C19 -> C18	Malignant neoplasm of the rectosigmoid junction	Malignant neoplasm of the colon	0.15%	70.00%	9.69
83	C19 -> C20	Malignant neoplasm of the rectosigmoid junction	Malignant neoplasm of the rectum	0.15%	70.00%	9.78
84	I10, I74 -> I63	Essential (primary) hypertension arterial embolism and thrombosis	Cerebral infarction	0.24%	70.00%	1.06
85	E77, E02 -> E11	Disorders of glycoprotein metabolism subclinical iodine-deficiency hypothyroidism	Type 2 diabetes mellitus	0.17%	69.70%	1.03
86	F80 -> F84	Specified developmental disorders of speech and language	Pervasive developmental disorders	24.88%	69.08%	2.56
87	K65, K80 -> K74	Peritonitis and cholelithiasis	Fibrosis and cirrhosis of the liver	0.49%	68.75%	4.99
88	I80, I25 -> I63	Phlebitis and thrombophlebitis chronic ischaemic heart disease	Cerebral infarction	0.27%	68.00%	1.03
89	I10 -> I63	Essential (primary) hypertension	Cerebral infarction	48.68%	67.92%	1.03
90	K70 -> K74	Alcoholic liver disease	Fibrosis and cirrhosis of the liver	2.57%	67.64%	4.91
91	S32, S02 -> S22	Fracture of the lumbar spine and pelvis and fracture of the skull and facial bones	Fracture of the rib(s), sternum, and thoracic spine	2.12%	66.67%	1.96
92	J03, J40 -> J18	Acute tonsillitis and bronchitis, not specified as acute or chronic	Pneumonia, organism unspecified	0.77%	65.57%	1.17
93	K25 -> K29	Gastric ulcer	Gastritis and duodenitis	2.88%	64.68%	1.21
94	K58 -> K29	Irritable bowel syndrome	Gastritis and duodenitis	0.71%	64.65%	1.21
95	K65 -> K74	Peritonitis	Fibrosis and cirrhosis of the liver	2.98%	62.41%	4.53
96	K57 -> K29	Diverticular disease of the intestine	Gastritis and duodenitis	1.25%	62.15%	1.16
97	J20 -> J18	Acute bronchitis	Pneumonia, organism unspecified	6.98%	62.11%	1.11

## Data Availability

All data are included in the manuscript. If needed, authors can provide the anonymous dataset.
